# Optimization of Liner Operations and Fuel Selection considering Emission Control Areas

**DOI:** 10.1155/2023/6351337

**Published:** 2023-07-07

**Authors:** Bin Yang, Jiahui Zou

**Affiliations:** Institute of Logistics Science and Engineering, Shanghai Maritime University, Shanghai 201306, China

## Abstract

The continuous expansion of shipping trade has brought about increasingly serious marine pollution problems. In the context of emission reduction in the global shipping industry, this paper focuses on the operation optimization of container ships inside and outside the emission control area (ECA). From the dual perspectives of shipowners and the general public, models in the annual operating cycle are established to study the economic and environmental benefit differences between traditional fuels, i.e., heavy fuel oil (HFO) and low-sulfur fuel oil (LSFO), and alternative fuels, i.e., liquefied natural gas (LNG) and methanol. Sensitivity analysis was carried out for the proportion of ECA and ship speed. The results show that, in the current situation of high natural gas prices, the use of HFO after the installation of scrubbers is still the most cost-effective option in the short term, followed by the use of LSFO and methanol. LNG is no longer an attractive option, while LSFO and methanol are the best options for both cost and the environment. With the tightening of ECA regulations, methanol will become the optimal choice when the ECA ratio is higher than 47%. By reducing the speed of the ship, the pollutant emission can be effectively reduced, but it will also lead to an overall decrease in profits. Considering the future “zero carbon” emission targets, slow streaming is only suitable as a short-term response measure, while switching to green power energy is a choice that is more in line with the long-term development strategy.

## 1. Introduction

International shipping, which serves as the main conduit for products moving across borders, transports more than 90% of goods traded globally and has made a great contribution to the growth of the world economy. However, due to the diverse, protracted, and flexible nature of ship transportation activities, the resulting large amount of air pollutants will cause serious environmental pollution in ports and coastal areas [1]. In 2018, the total emissions of the international shipping industry reached 1.056 billion tons of carbon dioxide equivalent, accounting for about 2.89% of the annual greenhouse gas emissions [2]. If no measures are taken, the total emissions are projected to increase by 50% to 250% in 2050 [3].

In this context, as the main governance bodies, various international organizations and sovereign countries have successively issued relevant policies to limit emissions from the shipping industry. The International Maritime Organization (IMO) has been dedicated to reducing carbon emissions in the global shipping sector since 2011. The most influential one is the MARPOL 73/78 Convention, which has been ratified by more than 160 countries. The convention includes six technical annexes, each of which contains detailed provisions on specific categories of pollution from ships. Among them, Annex VI imposes restrictions on the emission of pollutants such as nitrogen oxides (NOx), sulfur oxides (SOx), and greenhouse gases (GHGs) [4]. IMO has also set the Baltic Sea, the North Sea, North America, and the Caribbean Sea as emission control areas (ECAs), stipulating that from January 1, 2020, the global sulfur limit for ships' fuel oil will be reduced from 3.5% to 0.5%, while the upper limit within the ECA will be reduced from 0.5% to 0.1%, which are clearly listed in Table 1.

In addition, there is intense pressure on the shipping sector to reduce carbon emissions. With an initial strategy to reduce greenhouse gas emissions from ships, the IMO's Marine Environment Protection Committee has ambitiously joined the global quest for a path to decarbonization, with the following vision: International shipping's carbon intensity will decrease by at least 40% by 2030 compared to 2008, with a goal of decreasing by 70% by 2050. By 2050, the greenhouse gas emissions from international shipping will be reduced by at least 50% compared with 2008 and will reach the peak of emissions [5]. At the same time, the Chinese government also formally put forward the carbon peaking and carbon neutrality goals at the United Nations General Assembly in September 2020, striving to achieve carbon peak by 2030 and carbon neutrality by 2060 [6]. Under such increasingly stringent emission requirements, it is of great significance to study the choice of fuels in the context of dividing ECA. In order to provide a reference for the decision-making of various stakeholders and to some extent encourage the sustainable development of the global shipping sector, this paper evaluates alternative fuels with both economic and environmental benefits.

The rest of the article is organized as follows: Section 2 lists the current major emission reduction measures in the shipping industry and introduces several major types of exhaust gas after-treatment technologies and common marine fuels.  Section 3 establishes a mathematical model of pollutant emissions, private costs, and social costs of different fuels in the annual operating cycle from the dual perspectives of shipowners and the public.  Section 4 selects a specific route to conduct an example analysis.  Section 5 shows a sensitivity analysis conducted on the proportion of emission control areas and the speed of ships.  Section 6 summarizes the paper and provides a set of concluding remarks.

## 2. Emission Reduction Measures

As the global climate continues to deteriorate, the corresponding emission reduction policies are gradually tightening, and the operations of shipping companies will be directly affected. Currently, the methods to deal with emission restrictions mainly include four types: improving technical design, optimizing operation methods, using green power energy, and introducing market mechanisms.

Technical design measures are primarily aimed at improving the hull design and optimizing the engine system, such as the bulbous bow hull design, waste heat recovery system, and exhaust gas after-treatment device so as to maximize propulsion efficiency and reduce pollutant emissions. Among them, exhaust after-treatment devices mainly include scrubbers and selective catalytic reduction (SCR) devices, which can significantly reduce NOx and SOx emissions with little impact on engine performance and fuel economy [7]. SCR technology can achieve 90%–95% NOx reduction [8, 9], making it the most efficient NOx emission reduction method, while the desulfurization efficiency of scrubbers can be as high as 97% [10], allowing ships to continue to use heavy fuel oil (HFO). Scrubbers remain an attractive emission reduction option for shipowners given the current high price trends for low-sulfur fuel oil (LSFO) and liquefied natural gas (LNG). Some studies have comparatively evaluated the economic and environmental benefits of installing after-treatment devices and fuel-switching measures on ships [11–14], as well as changes in options as factors such as fuel prices [15, 16], emission regulations [17], and government subsidies [18].

The improvement measures of the operation plan primarily include the optimization of navigation routes, speed, fuel replenishment strategy, and fleet structure. Many researchers have conducted studies from various perspectives and have extensively verified the effectiveness of the deceleration ship scheduling method [19–21].

Low-carbon fuel is an effective way to reduce the carbon footprint, and zero-carbon fuel may be the main means to achieve carbon neutrality. Alternative fuels that have been considered in the research mainly include LNG, methanol, hydrogen, ammonia, liquefied biogas, and biofuels. In addition, a series of green power systems such as fuel cells, wind energy, solar energy, and nuclear energy have been gradually developed [22]. Although the most important fuel for shipping is still HFO, more and more shipowners have chosen to install or reserve alternative fuel systems for new buildings. In the first quarter of 2022, a total of 61% of the total tonnage of newbuilding orders can use alternative fuels, of which 57% of the orders use LNG fuel and 3.4% of the orders use methanol fuel [23]. Compared with traditional marine fuels, the carbon emission reduction potential of LNG and methanol is about 20%–40% [24–26], and the overall potential of alternative fuels to reduce SOx and NOx emissions can reach 60–90% and 80–85%, respectively [9, 26]. In addition, market mechanisms such as carbon tax and carbon trading can achieve the purpose of restriction by increasing the cost of carbon emissions, which will become one of the important ways for the low-carbon governance in the future.

Based on the above research, this study comprehensively considers the newbuilding orders in recent years and the physical and chemical properties of different fuels (see Table 2), retains HFO, MGO, and VLSFO as traditional fuel options, and selects LNG and methanol as alternative fuel options. Taking the following four emission reduction measures as evaluation scenarios, a mathematical model was established innovatively from the dual perspectives of shipowners and the public, and the annual pollution emissions and costs of various fuel-powered container ships were calculated, evaluating their economic and environmental benefits.

  Scenario 1: MGO (0.1%) and HFO (3.5%) are used inside and outside the ECA, respectively, and scrubbers and SCR equipment are used throughout
  Scenario 2: MGO (0.1%) and VLSFO (0.5%) are used inside and outside the ECA, respectively, using SCR equipment throughout
  Scenario 3: LNG is used as power throughout the process, and SCR equipment is used
  Scenario 4: methanol is used as power throughout the process, and SCR equipment is used

## 3. Mathematical Model

The model established in this paper is based on the following assumptions:

1. The auxiliary engine uses MGO throughout the process and does not switch with the main engine fuel.
2. The cost of new container ships for LNG and methanol is 20% and 15% [35] higher than that of traditional fuel ships, respectively
3. The ratio of the ship to the sailing mode and the port berthing mode is 9 : 1 [36], and the average speed in the sailing mode is 18 knots
4. In order to meet the strict NOx emission requirements, SCR equipment is required to be used throughout the process in all scenarios
5. The average service life of ships and SCR equipment is 25 years, and the average service life of scrubbers is 15 years [37]

### 3.1. Fuel Consumption

The fuel consumption of the ship is estimated by dividing it into two operating modes: sailing and port berthing. The main engine load in the sailing mode is the cubic ratio of the actual speed and the design speed, while the auxiliary engine load is generally considered to be independent of speed, and the value in this paper is 0.5 [38]. In the port berthing mode, only one auxiliary engine is reserved. The fuel consumption of the main and auxiliary engines is calculated by

(1) $$\begin{array}{c} F_{M}={SFOC}_{M}\times {EL}_{M}\times P_{M}^{design}\times 10^{-6}\text{,}\\ F_{A}={SFOC}_{A}\times {EL}_{A}\times P_{A}^{design}\times 10^{-6}\text{,} \end{array}$$

where *F*_*M*_ and *F*_*A*_ are the fuel consumption rate (t/h) of the main and auxiliary engines per unit time, respectively, when the ship is sailing; SFOC_*M*_ and SFOC_*A*_ are the specific fuel consumption factors (g/kWh) of the main and auxiliary engines, respectively; according to the existing research, this paper takes 196 g HFO/kWh and 216.7 g MGO/kWh, respectively [39]; EL_*M*_ and EL_*A*_ are the load factors of the main and auxiliary engines respectively; and *P*_*M*_^design^ and *P*_*A*_^design^ are the design rated power (kW) of the main engine and the auxiliary engine, respectively.

When using MGO and HFO inside and outside the ECA, respectively, the fuel oil consumed throughout the voyage is calculated as follows:

(2) $$\begin{array}{c} F_{HFO}=F_{M}\times \frac{D_{O}}{V}\text{,}\\ F_{MGO}^{M}=F_{M}\times \frac{D_{I}}{V}\times \frac{{LHV}_{HFO}}{{LHV}_{MGO}}\text{,}\\ F_{MGO}^{A}=n_{A}{\times F}_{A}\times \frac{D}{V}+\frac{1}{9}\times F_{A}\times \frac{D}{V}\text{,}\\ F_{MGO}=F_{MGO}^{M}+F_{MGO}^{A}\text{,} \end{array}$$

where *F*_HFO_ and *F*_MGO_ are the total consumption (*t*) of HFO and MGO, respectively; *F*_MGO_^*M*^ and *F*_MGO_^*A*^ are the MGO consumption (*t*) of the main and auxiliary engines, respectively, and the sum of the two is the total consumption of MGO; *V*_*d*_ is the ship's design speed and *V* is the actual sailing speed (kn); *D*_*I*_ and *D*_*O*_ are the sailing distance (n mile) of the ship inside and outside the ECA, respectively, while *D* is the total sailing distance (n mile); *n*_*A*_ is the number of auxiliary engines; and LHV_HFO_ and LHV_MGO_ are the low heating value (kJ/kg) of HFO and MGO, respectively, which can be used to convert the mass of different fuels under the same heat release.

Similarly, when VLSFO is used outside the ECA, the MGO consumption remains unchanged, and the fuel consumption of VLSFO can be expressed as

(3) $$\begin{array}{c} F_{VLS}=F_{HFO}\times \frac{{LHV}_{HFO}}{{LHV}_{VLS}}\text{.} \end{array}$$

When using alternative fuels such as LNG or methanol, MGO consumed by the auxiliary engines remains unchanged, and the fuel consumption of the main engine can be expressed as

(4) $$\begin{array}{c} F_{ALT}=F_{HFO}\times \frac{{LHV}_{HFO}}{{LHV}_{ALT}}+F_{MGO}^{M}\times \frac{{LHV}_{MGO}}{{LHV}_{ALT}}\text{,} \end{array}$$

where *F*_VLS_ and *F*_ALT_ are the consumption of VLSFO and alternative fuel (LNG or methanol), respectively (t), and LHV_VLS_ and LHV_ALT_ are the low heating value (kJ/kg) of the corresponding fuel.

### 3.2. Pollutant Emissions

The ten pollutant emissions reported by the IMO include CO_2_, CH_4_, N_2_O, CO, SOx, NOx, PM, NMVOC, and BC [2]. This paper selects three main greenhouse gases CO_2_, CH_4_, and N_2_O and three atmospheric pollutants SOx, NOx, and PM as emissions for quantitative evaluation. Pollutant emissions are represented by the product of fuel consumption and the corresponding emission factor, namely,

(5) $$\begin{array}{c} E_{ij}=F_{j}\times {LHV}_{j}\times {EF}_{i}\times 10^{-6}\text{,} \end{array}$$

where *E*_*ij*_ is the mass (t) of the emission *i* produced by the combustion of the fuel *j*, *F*_*j*_ is the consumption (t) of the fuel *j*, LHV_*j*_ is the low heating value of the fuel *j* (kJ/kg), and EF_*ij*_ is the emission factor (g/MJ) for the emission *i* of the fuel *j*. This paper assumes that the use of SCR and scrubbers can reduce NOx and SOx emissions by 90% and 95%, respectively. In addition, due to the limitations of current research on alternative fuels, some emission factors for methanol are not available. Since methanol does not contain nitrogen oxides and sulfur, we assumed that this part of the emissions is zero in the subsequent calculation. The emission factors for various fuels are shown in Table 3.

### 3.3. Annual Cost and Profit

The number of ships operating on a route in a year can be expressed as

(6) $$\begin{array}{c} n={\left[\frac{\left(365\times 24\times 9\times V\right)}{10}\times D\right]}_{Floor}\text{,} \end{array}$$

where the mathematical symbol []_Floor_ means the floor function. The costs involved in the operation of ships mainly include three parts: capital cost, operating cost, and fuel cost. The capital cost mainly includes the construction and installation cost of the new building and related equipment. Generally, the depreciation method of the average service life of the ship is adopted; i.e., the total investment cost is divided by the service life. The operating costs are the costs incurred by shipping companies to maintain normal shipping services, including equipment operating costs, crew wages, maintenance costs, and insurance and management fees, and port fees, loading and unloading fees, anchoring fees, etc., are generally 15%–50% of the capital cost [45, 46], and the compromise value in this paper is 30%. The fuel cost is affected by various conditions such as ship size, speed, and fuel and can be expressed as the product of fuel consumption, price, and number of sailings. For shipowners, the choice of an emission reduction plan mainly depends on the trade-off between capital expenditure (CAPEX) and operating expenditure (OPEX) [47].

The private cost and its subdivision cost ($) can be calculated as

(7) $$\begin{array}{c} PC={C_{FUEL}+C}_{CAPEX}+C_{OPEX}\text{,}\\ C_{FUEL}=\left(\underset{i}{\sum }F\times P\right)\times n\text{,}\\ C_{CAPEX}=\left(\frac{C_{ship}+C_{SCR}}{25}+i\times \frac{C_{scrubber}}{15}\right)\text{,}\\ C_{OPEX}=30\%\times C_{CAPEX}+\left(8\%+s\times 2\%\right)\times C_{FUEL}\text{,} \end{array}$$

where PC is the private cost of the shipping company, *C*_FUEL_ is the fuel cost, and *C*_CAPEX_ and *C*_OPEX_ are the capital cost and operating cost, respectively, which can be seen in Table 4; *C*_ship_ and *C*_scrubber_ are the investment cost of the new building and scrubber, respectively; *F* and *P* are the annual consumption (t) and price of the fuel ($/t); *s* is a 0-1 variable; if 0 is taken, it means that the scrubber does not need to be installed in this scenario, and if 1 is taken, it means that the scrubber needs to be installed.

The net profit of a single voyage can be expressed as the difference between the total revenue and the total private cost:

(8) $$\begin{array}{c} P=n\times r\times CL\times FR-C\text{,} \end{array}$$

where *n* is the number of voyages in one year as required above, CL is the container ship's load capacity (TEU), and *r* is the utilization rate of the space. In the situation where it is difficult to get one cabin, this paper takes the value of 1. According to the statistics of USDA [50], we take the average freight for all kinds (FAK) in the first half of this year as 1270 $/TEU.

### 3.4. Social Cost

Under the same conditions, shipowners and the public tend to prefer different optimal emission reduction options. Driven by economic interests, shipowners usually only pay attention to the private cost when they choose schemes, and their goal is to maximize the total profits on the basis of meeting the minimum emission requirements, while for the public, they are more concerned about whether the option reaches the best balance between economy and environment. Therefore, they need to consider the social cost of emissions, which can be expressed as the sum of the emissions of various pollutants multiplied by the corresponding cost factors:

(9) $$\begin{array}{c} SC=\underset{j}{\sum }\underset{i}{\sum }E_{ij}\times {CF}_{ij}\text{,} \end{array}$$

where SC is the social cost ($), *E*_*ij*_ is the emission *i* of the fuel *j* calculated above (t), and CF_*ij*_ is the social cost factor for the emission *i* of the fuel *j* ($/t). The social cost factors of different pollutants are shown in Table 5.

## 4. Case Analysis

### 4.1. Parameter Value

This paper selects the Northeast Asia-Australia route (A3N) operated by COSCO Shipping as an example. The route departs from Yokohama Port, goes through Osaka, Busan, Qingdao, Shanghai, and Kaohsiung Port, stops at Melbourne Port, and returns via Sydney Port and Brisbane Port and finally returns to the starting port of Yokohama Port, completing a round-trip voyage with a total sailing distance of about 13740 n miles. This paper only considers the countries and regions that have clearly divided the ECA; based on the longitude and latitude of the port and the reference point along the ECA, the total sailing distance within the ECA is calculated to be about 720 n miles. According to the latest shipping schedule released by COSCO Shipping, it can be seen that the operating ships of this route are post-Panamax container ships. The relevant parameters are shown in Table 6.

In 2020, the average price of LNG will remain around 400$/t, which is about 80% of the price of MGO fuel. Compared with expensive low-sulfur fuel, LNG has great price advantage and is considered to be a better emission reduction solution than other fuels in terms of economic and environmental effect [35, 43]. However, since the second half of 2021, the market price of natural gas has risen rapidly and the supply has become tight, and the conflict between Russia and Ukraine in 2022 further exacerbated this trend. Within a year and a half, the average price of LNG has risen to four times the original price, and the peak price even reached more than 3,000 $/t. At these prices, it is worth considering whether LNG ships are still a credible option to reduce emissions.

Based on the statistics of Ship & Bunker, this paper takes the average price of HFO, VLSFO, MGO, and LNG in Rotterdam Port from January to June 2022 as the benchmark price, which are 664, 884, 1120, and 1783 $/t, respectively; based on the statistical data of Methanex, this paper takes the mean value of the nondiscounted reference price of methanol in the same time period as the benchmark price, i.e., 630 $/t, and substitutes it into the mathematical model established above.

### 4.2. Pollutant Emissions

As can be seen from Figure 1, before the application of exhaust after-treatment equipment, the emission of pollutants from alternative fuels is significantly lower than that of traditional fuels. However, it is worth noting that when LNG is used as fuel, there is serious methane leakage, and the methane emission can be nearly 300 times that of ordinary fuel oil and more than 1000 times that of alternative clean fuels. Therefore, LNG may not be an effective scheme to mitigate climate change under comprehensive consideration.

Compared with HFO, alternative fuels can reduce SOx emissions by more than 99%, but the CO_2_ emissions of LNG and methanol do not have obvious advantages compared with traditional fuels. After switching to LNG and methanol, CO_2_ emissions can only be reduced by about 21.7% and 7.5%, respectively. After the application of scrubbers and SCR equipment, the SOx and NOx emission levels of traditional fuels are reduced to the emission range of alternative fuels, which is an effective emission reduction measure. Therefore, for shipowners, the choice of the best emission reduction scheme will depend on the trade-off between the installation and operating costs of different emission reduction equipment and the cost of switching fuel.

### 4.3. Cost

For shipowners, when making the choice of the best emission reduction scheme, the ultimate reference is the private cost. It can be seen from Figure 2 that, due to the absolute advantage of traditional fuel oil in price, the use of MGO and HFO inside and outside the ECA, respectively, is still the best choice for shipowners under the condition that exhaust after-treatment equipment is installed to meet the emission requirements, followed by the use of MGO and VLSFO inside and outside the ECA and the use of methanol. The skyrocketing price of LNG makes it no longer an attractive option.

When making decisions, the public should comprehensively consider private costs and social costs and make choices that have both economic and environmental benefits. It can be seen that the best solution at present is to use MGO and VLSFO inside and outside the ECA, followed by methanol as power. LNG can gain cost advantages over VLSFO only when the price drops by more than 40% and can obtain comprehensive advantages over methanol and VLSFO when the price drops by about 14 and 30%, respectively, which may not be possible in the short term.

## 5. Sensitivity Analysis

### 5.1. Ratio of ECA

More and more countries and regions have begun to divide the ECA and expand the scope of the existing ECA. With the increasingly tightened emission regulations, it is necessary to consider the impact of the proportion of ECA on emission reduction options. This paper calculates the changes in pollutant emissions, costs, and benefits when the time proportion of ships sailing in ECA increases from 2% to 20% in increments of 2%. Since both LNG and methanol are used in the whole process, the ratio of ECA has no effect on them. Meanwhile, the change in the ECA proportion has no impact on the single voyage time of the ship, so the total operating income remains the same, and the scheme with the lowest private cost is the scheme with the highest profit.

In terms of private costs, traditional fuel has great advantages. As shown in Figure 3, the use of MGO and HFO inside and outside the ECA, respectively, is the best choice, regardless of the proportion of the ECA. But after considering the social cost, when the proportion of the ECA is less than 46%, the best choice is VLSFO, methanol, and HFO in turn. When it is higher than 47%, methanol will be the best choice, followed by VLSFO and HFO, but when it rises to 58%, HFO will become better than VLSFO. Only when the proportion of the ECA is greater than 82%, LNG can have certain advantages over VLSFO, but the cost is still far higher than that of methanol. However, if VLSFO ships are also equipped with scrubbers, the environmental benefits will far exceed the investment and operating costs of scrubbers, and it will always be the best choice for shipowners when the ECA ratio is not more than 85%.

Extending this conclusion to other ships, it can be seen that if a container ship of the same size carries out short-range ocean transportation, when the proportion of its sailing in ECA exceeds 46%, it can be considered switching to use methanol as power. When the proportion is less than 85%, using VLSFO on the basis of adding scrubbers will bring the greatest profit.

### 5.2. Speed

In order to see the impact of speed on operating costs and emissions more intuitively, the range of speed is set to be 12–20 knots, and the pollutant emissions and costs are calculated separately. As the speed decreases, the load of the ship's engine gradually decreases, the corresponding fuel consumption and the emission of various pollutants will be reduced, and the overall fuel cost and operating cost of the corresponding solutions will drop. Under the condition of constant investment cost, both private and social costs show a decreasing trend. However, due to the decrease in speed, the operating voyages in one year will be reduced, and the annual profit at different speeds is shown in Figure 4.

Under the balance between the reduction of voyage benefits and the reduction of private costs, although the overall profit shows a gradual downward trend, there is an optimal speed in each speed segment, which enables the shipowner to obtain the highest profit, which is about 18.9 knots, 15.7 knots, and 12.6 knots, of which 18.9 knots can be used to maximize profits.

For the public, after taking the emission cost into consideration, it can be seen from Figure 5 that VLSFO is the most economical and environmentally beneficial choice at different speeds. When the speed is greater than 14 knots, methanol is the second-best choice; but with the decrease in speed, the price advantage of HFO will be more prominent, and its total cost will be lower than that of methanol.

## 6. Conclusion

Shipowners must consider different emission reduction solutions when placing orders for new ships in order to comply with increasingly stringent international conventions and regulations, including continuing to use HFO after adding scrubbers and switching to low-sulfur fuel oil and cleaner alternative fuels such as LNG and methanol.

This paper assesses the pollutant emissions of various fuels in the annual operation cycle of ships, taking into account both the economic and environmental benefits. A private and social cost model was developed to assess the best mitigation options in the context of current fuel prices. The study takes into account how compliance decisions made by shipowners and the general public alter under various ECA ratios and speed situations, and the following results are drawn:

1. VLSFO, LNG, and methanol can effectively reduce SOx emissions by more than 90% compared with HFO, but LSFO and methanol can only reduce CO_2_ emissions by 2% and 8%, respectively, and have no obvious advantages in CO_2_ emission reduction.
2. The most economical option at the moment is to continue using HFO after installing scrubbers, but converting to LSFO will be preferable when taking into account the social cost of emissions.
3. When the ECA ratio is greater than 47%, methanol will become the best choice for both the environment and the cost. At the same time, reducing the speed of sailing is indeed one of the effective measures to reduce emissions in the short term, although it will reduce the annual profit.

The service life of ships is often between 20 and 30 years, and the choice of a power system will have a long-term impact on the future environmental climate. Considering the number of new ship orders, we focused on container ships as research objects, but similar methods can be extended to other ship types, such as dry bulk carriers and oil tankers, providing useful reference for various stakeholders to make dynamic decisions through horizontal comparisons, reduce cost, and maintain market competitiveness in the context of tightening environmental policies and changing fuel prices. In addition, it should be pointed out that this paper substitutes the historical average data of fuel prices into the calculation, but considering the instantaneous changes in fuel prices, it will be possible to update fuel prices, fuel consumption, and other parameters in real time and expand the existing model into a dynamic decision-making model in the next step.

When it comes to choosing a long-term sustainable alternative fuel, there is no single answer as to which is the best choice. It is determined by a number of elements, including various operation modes, the scope of ECA laws, and the principal authority making the decision. However, it is apparent that the transition to cleaner and more efficient fuels will be an unavoidable trend in the future.

## Figures and Tables

**Figure 1:** Pollutant emissions of different options.

**Figure 2:** Cost of container ships under different options.

**Figure 3:** Private cost and total cost under different ratios of ECA.

**Figure 4:** Annual profit at different speeds.

**Figure 5:** Total cost at different speeds.

**Table 1:** Restrictions on sulfur content of marine fuels in MARPOL Annex VI.

Global sulfur limit	Emission control area
4.50% prior to January 1, 2012	1.50% prior to July 1, 2010
3.50% on and after January 1, 2012	1.00% on and after July 1, 2010
0.50% on and after January 1, 2020	0.10% on and after January 1, 2015

**Table 2:** Physicochemical properties of different fuels.

	HFO	MGO	VLSFO	LNG	Methanol
Storage form	Liquid	Liquid	Liquid	Cryogenic liquid	Liquid
Pressure, temperature (bar, °C)	1, 25	1, 25	1, 25	1, −162	1, 25
Liquid density (kg/m^3^)	986–1010	855–860	975–1010	430–470	790–792
Lower heating value (kJ/kg)	40200	42800	40500	48600	20000
Energy density (kJ/L)	39100	35800	36400	20800	18200

^*∗*^Data source: summarized from the recent literature [4, 27–34].

**Table 3:** Emission factors for different fuels.

	HFO	MGO	VLSFO	LNG	Methanol
CO_2_	77	75	74	54	69
CH_4_	0.0015	0.00142	0.00143	0.562	N/A
N_2_O	0.004	0.003738	0.00357	0.00463	N/A
SOx	1.277	0.0467	0.2347	0.00056	N/A
NOx	1.532	0.483	0.483	0.1611	0.28
PM	0.1811	0.0227	0.1014	0.0037	0.0043

^*∗*^Data source: summarized from the recent literature [10, 28, 40–44]. ^*∗∗*^N/A means data for that indicator are not available.

**Table 4:** CAPEX and OPEX for the scrubber and SCR equipment.

	CAPEX	OPEX
Scrubber (m$)	2.5–3 (open-loop)	1–3% of fuel cost
	4.5–5 (closed-loop)	

SCR ($/kW)	40–135	7–10% of fuel cost

^*∗*^Data source: summarized from the literature [48, 49].

**Table 5:** Social cost factors of different polluting gases [4].

Gas	Social cost factors $/T
CO_2_	56.6
CH_4_	1750
N_2_O	15000
SO_2_	24900
NOx	34700
PM	79500

**Table 6:** Sample vessel and engine parameters.

*Sample ship*				
Builder	TEU	DWT	Speed (kn)	Price (m$)
New Times SB	7000	81689	20	75.13

*Main engine*				
Model	Type	Bore/stroke	Power (kW)	Speed (rpm)
MAN B. & W. 7G80ME-C10.5	2-stroke 7-cyl	800 mm × 3720 mm	26280	72

*Auxiliary engine*				
Model	Type	Bore/stroke	Power*∗*number (kW)	rpm
HHI-EMD (HiMSEN) 8H32/40	4-stroke 8-cyl	320 mm × 400 mm	4000*∗*3	720

## Data Availability

The data used to support the findings of this study are included within the article.
